# Research on Organization Design of College Chinese Teaching under Big Data Environment

This article has been retracted.

**DOI:** 10.1155/2022/2774072

**Published:** 2022-08-18

**Authors:** Jiayu Shi, You Wu

**Affiliations:** ^1^Inner Mongolia Technical College of Mechanics and Electrics, Hohhot 010070, Inner Mongolia, China; ^2^Qiannan Normal University for Nationalities, Duyun 558000, Guizhou, China

## Abstract

The pivotal and most important technology point of the application of big data in modern network teaching is the establishment of teaching platform. Based on Hadoop big data technology, this paper establishes a big data platform designed by Chinese teaching institutions in colleges and universities. The teaching system not only realizes the diversified development of network teaching but also realizes the discovery of teaching platform users' needs and the push of resources. In addition, it is found that a small number of people do not have a high understanding of the teaching mode of big data through extensive studies, which also shows that traditional teaching is still lagging behind in big data education. However, on the whole, the Chinese teaching model in universities based on the big data environment deserves further promotion and application in universities.

## 1. Introduction

In recently years, as China's image as a major power is gradually recognized by the international community, China is playing an increasingly important role in the world's economic and cultural exchanges. As the mother tongue of China, learning Chinese has become an inevitable and irresistible trend of economic globalization. At the same time, we have also rapidly entered the era of big data with the rapid development of the Internet. The big data has had a significant impact on finance, business, medical care, and other fields [1, 2]. Accordingly, how to reasonably design or carry out Chinese teaching under the platform of big data is an important problem that restricts the development of the teaching level of the universities in China.

Some scholars gradually focus on the development and application of big data technology in the field of driving in recently years [3–19]. The US Department of Education was the first to release the education data mining and discussed the future development and application of big data in the field of education [3]. He et al. (2014) and Chen et al. (2014) had pointed out that the introduction of big data technology can promote the process of educational informatization and provided specific directions for scientific educational decision-making in the field of education. Timms (2016) proposed that the purpose of education big data environment is to provide a better teaching environment so that teachers and students can better participate in teaching. With the help of the development of computer technology, it has optimized and improved the modern teaching platform to a certain extent, thus creating a more suitable intelligent and highly integrated teaching environment. Brundage (2015) explored the integration of artificial intelligence and education and designed an intelligent teaching system that can simulate student learning, has wide applicability, and enables autonomous social connections with learners. Lv et al. (2015) designed and studied mathematics teaching programs with big data technology, constructed corresponding intelligent system, and verified the system with experimental research, providing theoretical reference for subsequent mathematics teaching reform. Li et al. (2015) proposed the reform measures of university teaching methods under the big data environment. Chen et al. (2022) deeply explored the relationship between artificial intelligence technology and English teaching and establish an online intelligent English learning system based on big data network. From the different perspectives of social background, college education, and teaching subject and object, Wang (2021) deeply discussed how to put forward new innovations in the teaching mode of piano group class and sought ways to cultivate the teaching ability of piano group class on this basis. Liu et al. (2021) attempted to establish a connection between artificial intelligence technology and college English teaching and analyzed the advantages of the English teaching model based on artificial intelligence technology. Lin et al. (2017) elaborated the problems faced by database courses for computer majors in the era of big data and probed into the reform strategies and measures of computer professional curriculum database in the big data environment from two different perspectives of theoretical and experimental teaching. To some extent, the above research has promoted the rapid development of relevant teaching fields in the big data environment and provided corresponding references for the expansion of big data platform in the teaching field. However, there are few researches on Chinese teaching in universities. Considering that Chinese plays an important role in people's daily life and even in international exchanges, it is very important to carry out research on the organization design of Chinese teaching in universities under the platform of big data.

Based on the above existing research, this paper establishes a teaching platform designed for Chinese teaching organization in universities under the environment of big data and gives full consideration to the student-centered teaching goal in the teaching design. Based on Hadoop big data technology, the platform quickly locates students' teaching resource needs through image recognition technology and further improves the accuracy of data mining through in-depth mining of teaching data. In order to underline the advantages of the big data teaching platform established in this paper, the corresponding traditional teaching template is set as a comparison. Meanwhile, the big data Chinese teaching mode is further improved by using research. The results show that the new teaching platform based on big data environment can better upgrade the quality of Chinese teaching in universities.

## 2. Teaching Mode in Universities under Big Data Environment

According to the statistics on the number of universities and students released by the Ministry of Education of China in 2016, the number of universities in China that ranked second in the world is 2,879, and the number of undergraduates reached 37 million, ranking first all over the world. However, it is worth noting that, under such a huge scale of education, most of China's higher education is far behind the world's average education level, and the main factors leading to this are reflected in the following. First, the traditional education concept is backward, and the teaching mode still adopts the traditional “didactic.” Second, there is no sufficient interaction between students and teachers, which makes teachers' teaching and students' learning in a full disjointed state [20]. Finally, the lack of modern teaching equipment or low level of maintenance is also a vital element.

The backwardness of teaching mode and concept is the main factor restricting the development of Chinese teaching in universities. Although many schools are actively popularizing modern teaching equipment, it is difficult to fundamentally improve the teaching quality by simply introducing equipment. It is very important to establish an intelligent Chinese teaching platform in colleges by using big data and Internet technology. On the one hand, the established big data environment platform can facilitate for students to perform Chinese culture learning and communication anytime and anywhere, and on the other hand, the students choose a wider range of teachers or courses. In addition, the organization design and research of Chinese teaching under the big data environment can not only boost the implementation of diversified teaching mode, innovate the way of talent training, and upgrade the reform of education and teaching, but also realize the comprehensive informatization of the teaching environment in universities, so as to further the teaching quality and management efficiency.

### 2.1. Introduction to Big Data Environment Platform

In the age of big data, Victor Mayer-Schonberg predicted that 2013 would be the first year of the age of big data, marking that the development of information technology has entered a new development era [21–23]. With the development of society, especially the emergence of the Internet and the rapid development of information technology such as smartphones, computers, and cloud computing in recent years, the data generated by society every day is exploding.  Figure 1 shows the annual scale of global data presented in data age 2025. The era of big data has changed the traditional learning mode in Chinese education. The students' information sources are no longer limited to textbooks, but more from computers or mobile phones and other electronic devices. The unprecedented and powerful development trend of big data is gradually subverting the development of Chinese teaching in colleges and universities, but it also provides corresponding opportunities for the reform and innovation of Chinese teaching system in colleges and universities.

### 2.2. The Change of College Traditional Teaching Mode

In the traditional didactic teaching mode, teachers make teaching decisions mainly through their own intuition [24]. This kind of solidified experiential attention teaching often makes teachers immerse themselves in the past teaching experience and ignore the teaching reform brought by the continuous development of the times. At the same time, the teachers are often unable to accurately analyze and summarize classroom feedback, which undoubtedly leads to the arbitrariness and procedural nature of teachers in teaching decision-making. The solidified teaching model leads teachers to stick to their own teaching decisions. Ignoring the difference between students' acceptance of knowledge often results in low learning efficiency of some students.

The traditional teaching decision-making often takes the teacher as the main body and neglects the student-centered teaching objective. The traditional teaching-centered decision-making often fails to accurately target each student's learning situation and is gradually questioned and abandoned due to the limitations of teacher selection in the traditional teaching mode, as shown in Figure 2. The student-centered teaching mode is gradually coming into the education area. However, how to implement this teaching decision needs to make use of the Internet and big data environment platform and constantly revise teaching methods and contents through the powerful data analysis and summary ability of big data. In addition, the establishment of the teaching platform in the big data environment also allows students to choose a diversified teacher, which can full play the student-centered teaching concept of the new era.

The students' learning is often in a passive state and the learning materials are relatively single under the traditional teaching mode. A lot of knowledge is difficult to understand and master only by reading books. Furthermore, books are not easy to carry. However, the era of big data is completely different. With the support of various terminal devices and information technology such as the Internet, learning materials are extremely rich. In addition to books and notes, there are e-books, online videos, online simulation experiments, and so on. Students can read any knowledge they want through their mobile phones. Students are no longer limited by heavy books, so that learning becomes active. Moreover, video and online simulation experiments are more conducive to students' grasp and understanding of knowledge and help to stimulate students' enthusiasm in pursuing knowledge. This is a great boost to students' learning and can help students better grasp the course knowledge. In short, facing the arrival of the era of big data, teachers still use hardened experience to make teaching decisions, which will lead to teachers unable to accurately grasp the difficulty of teaching and the change of learning situation. Correspondingly, it will also lead to difficulties for teachers to provide effective guidance for subject teaching.

## 3. Technical Elements of Big Data Environment Platform Design

The design of college Chinese teaching platform is based on cloud computing hierarchical service framework, which collects, integrates, and analyzes various teaching data. Through big data integration technology, the connotation relationship of Chinese teaching is mined, and the content of Chinese teaching in colleges and universities is realized based on personalized recommendation. The platform can provide users with active course selection, learning and other services, with cultural content subscription, book retrieval and download, video on demand, visual image recognition, and other functions. The construction of the big data environment platform for college Chinese teaching can timely obtain the relevant learning information of students on the online learning platform. Using data analysis technology to analyze this information, mining students' learning behaviour characteristics, learning hobbies, learning objectives, development direction, and knowledge has been mastered, etc. Grasp students' learning progress and learning situation in real time, and establish knowledge map for students. Then, personalized guidance, recommendation, and suggestions are given to students according to the knowledge graph to realize intelligent teaching, so as to solve the problems that students actually need.

Figure 3 shows the overall framework of big data platform for Chinese teaching in universities. The big data platform of Chinese teaching in universities has realized the functions of data collection, data preprocessing, and big data storage and management. Teaching big data runs through preclass, in-class, and after-class in a whole-process and multidimensional way, integrating online and offline as well as in and out of class. Taking teaching data as bus, it serves teaching evaluation. The big data platform of Chinese teaching in colleges and universities mainly carries out teaching from three aspects, data collection and integration, data analysis and interpretation, and data application and early warning, and provides standard external data reading interface and graphical data management operation and maintenance. (1) Data acquisition and integration: colleges and universities can display and graphically collect different kinds of data in physical space, such as teaching platform data source, teaching environment data source, teaching supervision data source, and business system data source, providing comprehensive analysis results of big data with powerful real-time and offline computing capability. (2) Data analysis and interpretation: through data cleaning and deep machine learning, redundant data can be eliminated effectively, data structure can be optimized, efficient statistical analysis function can be realized, and intelligent data mining and data fusion can be carried out. (3) Data application and early warning: through the analysis of educational data, the big data analysis platform can deeply dig out students' learning behaviour and actual learning state during learning, such as accurate portrait analysis, personalized learning push, intelligent generation of knowledge map, customized teaching data report, and other functions. It can be applied in teaching decision-making and other aspects to provide in-depth comprehensive analysis results of big data for Chinese teaching in colleges and universities, so as to build the foundation of mass data in-depth analysis for university users, mining the potential core value of data and assisting decision-making.

### 3.1. Hadoop Environment Construction

Hadoop distributed system framework can complete a highly reliable and scalable distributed open-source software project. The Hadoop is designed to handle very large data sets and provides the ability to handle large data sets [25]. In addition, it can not only realize the parallel access of big data, but also closely combine real-time database technology and relational database. However, the most commonly used computer system in China is Windows, while Hadoop only supports Linux. Therefore, you need to download Ubuntu, a common Linux operating system, and build a Hadoop environment on it.

### 3.2. Database Technology

The teaching data of Chinese teaching platform in colleges and universities should be stored, updated, queried, downloaded, and transmitted. This system uses SQL statement to construct database management subsystem using server database technology. SQL server is a relational database management platform, which can provide more secure storage functions and has good flexibility and integration [26]. In the process of building this system, SQL server technology is used to build a B/S architecture model system. The system can not only quickly analyze data sources, but also have the ability of online data analysis and data mining. The online analysis and processing function enables the system to exchange information with other hosts within the scope of Internet and LAN and obtain diversified big data teaching platform resources. Data mining function is an advanced process of extracting potential, effective and understandable patterns from massive data according to the established goal, which can provide corresponding data processing, analysis work, and facilitate the identification and rapid positioning of teaching resources for intelligent image recognition.

In order to carry out data mining more efficiently, mining interference data sources can effectively improve the accuracy of data. Before efficiently mining data estimators, it is necessary to analyze the characteristics of big data parameters. Select student data in SQL database, on the basis of a large number of differential characteristic data, set the whole data estimator set *A*={*P*, *Q*}. *P* and *Q* are the first half and the second half of the data estimator, respectively. Since the data characteristics of different servers vary greatly, it is assumed that the data in the first half of the whole data set have *p* species parameter characteristic changes, and the data in the second half have *q* species parameter characteristic changes:

(1) $$\begin{array}{c} P=\left\{m_{1},m_{2},m_{3},\ldots ,m_{p-1},m_{p}\right\},\\ Q=\left\{n_{1},n_{2},n_{3},\ldots ,n_{q-1},n_{q}\right\}, \end{array}$$

where *m*_*i*_ and *n*_*j*_ are, respectively, the data curve fitting and result and line fitting results in a certain period, and 1 ≤ *i* ≤ *p*, 1 ≤ *j* ≤ *q*.

The set of data estimators covers a lot of information, so it needs to rely on big data analysis technology to achieve the set analysis. Big data analysis technology can refine the data interval and mine a large amount of valid information from the interval. Under big data analysis, curve fitting results *m*_*i*_ and linear fitting results *n*_*j*_ in a certain period of time have their own property variables *C* and proportion of variables *D*, namely,

(2) $$\begin{array}{c} m_{i}=\langle C_{i},D_{i}\rangle ,\\ n_{j}=\langle C_{j},D_{j}\rangle . \end{array}$$

In addition, the quantity of the nature variable and the proportion of the variable in the data estimator set are *p*+*q*, and ∑_*i*=1_^*p*+*q*^*D*_*i*_=1, and the set can be expressed as *G*={*m*_1_, *m*_2_, *m*_3_ ⋯ *m*_*p*−1_, *m*_*p*_, *n*_1_, *n*_2_, *n*_3_ ⋯ *n*_*q*−1_, *n*_*q*_}.

When selecting data sources in SQL database under big data environment, there will be some high noise interference data. The deviation of these data is large and will affect the accuracy of the model to some extent. Therefore, it is necessary to filter it effectively to ensure the correctness of the received data. When data deviation filtering is performed, two data point thresholds *M* and *N* need to be extracted, and the threshold of one data point needs to be larger. When 0 < *M* < *N* < 1 or 0 < *N* < *M* < 1, the similarity between the two data points can be determined. Big data clustering analysis clusters data into a class *l* reliable set *Z*_*l*_, including three kinds of data to be integrated, to be fitted, and to be filtered. If the parameter is met ‖*Y*_*j*_ − *Q*_*j*_‖ < ‖*Y*_*j*_ − *Q*_*t*_‖, it is the data to be integrated, that is, *Y*_*j*_ ∈ *M*.  Figure 4 shows the mining flow chart of interference data sources.

After deleting A from *Z*_*l*_ and writing *M*, the clustering center point of *Y*_*j*_ needs to be recalculated [27]. The corresponding function expression can be expressed as follows:

(3) $$\begin{array}{c} Q_{t}=\frac{1}{m_{k}}\sum Y_{j}^{x}\left(x=1,2,3\cdots K-1,K\right), \end{array}$$

where *m*_*k*_ is the number of data points in *Z*_*l*_; *x* is the number of big data clustering analysis layers; *t* is the amount of class *l* data.

In order to mine interference data more accurately, a threshold of mining accuracy can be set. When the mining accuracy is less than *χ*, (1) should be used for secondary mining [28]. The function expression of mining accuracy in the process of interference data mining can be given as follows:

(4) $$\begin{array}{c} f=\frac{1}{m_{k}}{\sum \left|Y_{j}^{x}-Q_{t}\right|}^{2}. \end{array}$$

### 3.3. Intelligent Identification Technology

In order to quickly process the corresponding data information in the teaching process after the user captures the video screenshot, this system uses convolutional neural network technology as the corresponding support. This technology is based on convolutional neural network, which can not only better adapt to the image structure but also carry out feature extraction and classification, making feature extraction conducive to feature classification. At the same time, the video screenshots captured by users are processed intelligently, and accurate matching queries are made on the large database platform. The collected pictures can be exchanged with the database resource information in this way.

## 4. Design of Big Data Environment Platform

### 4.1. Establish a Platform Framework

The teaching platform established in this paper under the big data environment is mainly supported by Hadoop technology. How to build the Hadoop framework will be explained later in this article. In order to facilitate the use of users, the platform uses Windows system as the front-end operating system. The Ubuntu system under the Hadoop architecture is used to simulate the big data teaching environment.

The system managers can easily manage and configure all node units in the cluster by operating the infrastructure module. In addition, managers can achieve further control over the cluster by creating and configuring an open-source project environment for big data analysis and management. In the big data infrastructure module, the cloud engine realizes the management of distributed Hadoop nodes through the task scheduling function. Meanwhile, other modules in the system, such as the database management module of video recognition, also need to adopt the task scheduling method to manage the database. Therefore, asynchronous mode is adopted for task transfer, which also ensures the rapid development and commissioning of submodules. The task script is developed in Python and consists of two parts, task and task fragment. Tasks are initialized to run on the administration server by reading in policy files. In addition, task scripts and shell scripts are packaged according to the corresponding configuration in the policy file. After the package is completed, it is sent to the proxy service module of Hadoop node through Socket. The proxy service module decompresses tasks and shell scripts to execute task fragment scripts. Then the corresponding shell script is invoked to complete the task scheduling and return the execution results to the cloud engine.

As shown in Table 1, real-time monitoring of the running status of Hadoop nodes, such as CPU usage, memory usage, QPS, and network status, is an important operation and maintenance method to guarantee the normal system operation. Combined with the characteristics of Hadoop node status monitoring, this paper developed the real-time node monitoring function based on open-source RRD (Round Robin Database) technology. RRD and its management agent are deployed on each Hadoop node. Real-time dynamic and static data of each node, such as task execution and node status, are reported to the cloud engine through the node monitoring plug-in. The cloud engine uses Memcashed technology to store node status information and is connected to the elastic scheduling module of the public cloud. When the Hadoop cluster load exceeds the specified threshold, the Hadoop cluster can be dynamically expanded or shrunk flexibly. The whole Hadoop big data teaching platform is set up as follows.

First, install and configure Ubuntu. Ubuntu is an interactive emulation environment that supports every version of Windows. In this environment, the front-end and back-end management of the platform can be realized. The installation and configuration process of Ubuntu is also very convenient. Simply go to the Ubuntu website, download the Ubuntu version for Windows, and click Install.

Second, install and configure Hadoop. Go to the official website to download and decompress the Hadoop installation package and then configure Hadoop. All configuration files are text files that can be edited using the vi editor or any text editor. Some XML configuration files use a uniform format, where each property node corresponds to a configuration, and there can be multiple configurations in a file. Finally, format HDFS.

### 4.2. Video Design

The main function of this system is the playback of teaching video courseware, so as to provide students with the most intuitive teaching experience and teaching visual impact. The specific implementation method is to take the B/S structure as the core of the organization, so that the basic functions of video can be realized more quickly, such as video uploading and downloading. The video sharing can be realized by means of modern teaching equipment in multimedia classrooms.

### 4.3. Data Collection

Database acquisition often uses SQL to store and collect data. The big data collection is accomplished by setting up a large number of databases at the collection end and carrying out load balancing and sharing among these databases. The perceptual device collection is mainly through the collection of video image information intercepted by the author, after the identification of the image information is collected in the database for storage.

### 4.4. System Accuracy Test

In order to test the basic performance of big data Chinese teaching, this paper selects data loss rate and transmission speed as the two basic detection indexes. The test results are shown in Table 2, which can observe that the data loss rate increases with the increase of data quantity. This is mainly because the corresponding interference data will also increase when the amount of data increases. However, the overall data loss rate is lower than 0.5%, which meets the basic requirement of data loss. In addition, the increase of data volume has no impact on the data transmission speed, and the current speed meets the basic requirements of the platform for real-time data.

## 5. Results

In order to emphasize the advantages of teaching mode based on big data platform compared with traditional Chinese teaching mode, two classes of students were randomly selected as the research objects. This paper analyzes the influence of different teaching modes on Chinese in colleges. The specific operation is that, in the whole semester, the experimental class and the control class adopt the teaching mode of big data platform and the traditional teaching mode, respectively. Students' monthly reading comprehension test scores and the final exam scores were summarized as the evaluation basis. The results are listed in Table 3 and Figure 4. From Table 3, the performance of the experimental class is better than that of the control version, and with the passage of time, the performance of the experimental class steadily improves. On the contrary, the performance of the control class is basically stable and obviously weaker than that of the experimental class. Similarly, the performance of the experimental class is significantly better than that of the control class in the final test from Figure 5. At the same time, the number of failed students in the experimental class was only 2, much lower than that in the control class. Compared with the final test scores of students in the control group, the scores of students in the experimental group are obviously better. All the above results well demonstrate that the teaching mode at the big data environment can give more play to students' subjective initiative and improve students' academic performance better than the traditional mode.

To further explore the acceptance of the college Chinese teaching model based on the big data platform among different groups, an online survey was conducted for 1,000 people in different universities. The investigated groups include students, teachers, teaching administrators, judges, and social staff, and the results are shown in Figure 6. The results from Figure 6 show that most people accept the teaching mode of Chinese in colleges and universities under the environment of big data, and about 20% of them think there is not much difference between the two teaching modes. In addition, about 10 percent think traditional teaching methods are better than big data ones. Through further sorting out the survey data, it is found that the main reason for this phenomenon is that most voters are nonstudents, who receive traditional didactic education and have less contact with the rapidly developing big data teaching model, so they cannot make reasonable evaluation.  Figure 7 lists the teaching evaluation chart adopted in this paper. After further summarizing the research results, feedback will be given to the big data teaching platform to further improve the recognition of the big data teaching model.

## 6. Discussion

### 6.1. Teaching Suggestions in Big Data Environment

In the environment of big data, teachers should not only rely on teaching experience and collective strength to form teaching decisions in teaching practice, but should rely more on scientific basis and teaching empirical research results to make decisions. After finding real problems in teaching through data analysis, teachers need to improve teaching strategies and solve real problems according to the actual situation of students. According to the content of data analysis and evaluation feedback, the teaching and research department of the school and teachers have full discussion and make teaching decision improvement plan. In the process of teaching decision implementation, the teaching and research group carries out tracking research through the data platform to ensure the improvement of teaching decision is effective. Regional schools gradually establish evaluation indicators based on the overall development of students, including school enrollment, school scale, school conditions, teacher level, and other factors. On this basis, schools rely on big data platform to promote scientific evaluation and further improve teachers' teaching decisions. The teaching evaluation supported by education big data integrates and analyzes students' learning background, learning process, and other data to provide personalized evaluation reports for students. On the basis of the big data platform, the scientific implementation of education and teaching evaluation mechanism based on problem diagnosis and guidance can help teachers timely discover real problems and conduct real research. In addition, teachers should make more reasonable education and teaching decision-making plan and real improvement and guide students to develop in an all-round way.

### 6.2. Learning Suggestions in Big Data Environment

The big data technology can easily transform students' learning behaviors into corresponding data for storage and recording. Therefore, as long as the state information in the learning process of students can be completely collected, the data can be analyzed and mined through big data or modeling methods. Then, the students' learning behavior and performance are evaluated and intervened according to the results, so as to predict the trend of students' future learning performance. More effective intervention methods and improvement measures can also be tailored for students to ensure their personalized development. It is necessary to implement the whole process of accurate teaching before, during, and after class to make students truly realize personalized learning. To achieve “accurate teaching,” we should conform to the learning situation and living situation. Teachers should rely on empirical evidence and data analysis to conduct in-depth interpretation and analysis in the aspects of accurate textbook interpretation, accurate goal setting, accurate classroom teaching, and accurate feedback evaluation. The above analysis results can guide teachers to improve teaching, optimize and reform teaching methods, and improve teaching quality.

## 7. Conclusion

With the rapid development of Internet and big data technology, network teaching mode has entered people's vision. Taking Hadoop technology as the core, this paper constructs a highly integrated Chinese teaching big data platform through in-depth data mining. Through the comparison with the traditional teaching mode, it is found that the big data teaching platform has better effect. In addition, through extensive research, it is also concluded that the popularity of big data teaching platform is better than that of traditional teaching mode. On this basis, the teaching and learning strategies based on big data teaching platform are proposed for teaching subjects and teaching objects. In general, the teaching platform has a strong promotion value.

## Figures and Tables

**Figure 1:** Gradual changes in global data volumes.

**Figure 2:** The difference between traditional teaching mode and big data teaching mode.

**Figure 3:** Overall framework of big data platform for Chinese teaching in colleges and universities.

**Figure 4:** Mining flow chart of interference data sources.

**Figure 5:** Final test score summary in different class.

**Figure 6:** Statistics on the results of extensive research on teaching model.

**Figure 7:** Teaching evaluation feedback diagram.

**Table 1:** Hadoop platform cluster configuration.

Server role	IP address	Node role	JDK version	Operating system
Master	192.168.03	NameNode	Java version	Windows
Slave1	192.168.04	DataNode	1.7.0_75	Ubuntu17.04
Slave2	192.168.05	DataNode	—	64 Bit

**Table 2:** Big data Chinese teaching platform test results.

Data size (G)	Loss rate (%)	Data processing rate (MB/s)
200	0.04	47.37
400	0.09	46.98
600	0.12	47.12
800	0.16	47.85
1000	0.21	47.56

**Table 3:** Monthly assessment results in different class.

Month	September			October			November		
Grades	O	G	*P*	O	G	*P*	O	G	*P*
Experimental class	29	24	7	30	25	5	32	26	2
Control class	20	28	12	21	29	12	19	28	13

O: outstanding (85–100); G: good (60–84); P: poor (0–59).

## Data Availability

The experimental data used to support the findings of this study are available from the corresponding author upon request.
